# The effect of synbiotic supplementation on atherogenic indices, hs-CRP, and malondialdehyde, as major CVD-related parameters, in women with gestational diabetes mellitus: a secondary data-analysis of a randomized double-blind, placebo-controlled study

**DOI:** 10.1186/s13098-022-00858-1

**Published:** 2022-06-21

**Authors:** Zohoor Nabhani, Cain C. T. Clark, Nazanin Goudarzi, Alemeh Hariri Far, Elham Razmpoosh

**Affiliations:** 1 Nutrition Research Center, Department of Biochemistry and Diet Therapy, Faculty of Nutrition and Food Sciences, Tabriz University of Medical Sciences, Tabriz, Iran; 2 Centre for Intelligent Healthcare, Coventry University, Coventry, CV1 5FB UK; 3 Department of Nutrition, Electronic Health and Statistics Surveillance Research Center, Science and Research Branch, Islamic Azad University, Tehran, Iran; 4 Integrative Oncology and Quality of life Department, Breast Cancer Research Centre, Motamed Cancer Institute, Academic Centre for Education, Culture, and research, ACECR, Tehran, Iran; 5 Department of Community Nutrition, Faculty of Nutrition, Tabriz University of Medical Sciences, Tabriz, Iran; 6 Nutrition and Endocrine Research Center, Research Institute for Endocrine Sciences, Shahid Beheshti University of Medical Sciences, Tehran, Iran

**Keywords:** Synbiotics, Diabetes, Gestational, Gestational, Atherogenic Index of Plasma, Malondialdehyde, C-Reactive protein

## Abstract

**Background:**

Women with GDM have a higher risk of future cardiovascular diseases (CVD). Meanwhile, synbiotics have been demonstrated to have favorable impacts on atherogenic indices, and inflammatory and oxidative stress indicators, all of which are known to be CVD-predictive factors. The aim of this randomized controlled trial was to evaluate the effects of synbiotic supplementation on the atherogenic indices of plasma, high-sensitivity C-reactive protein (hs-CRP), and plasma malondialdehyde (MDA) in women with GDM.

**Methods:**

Eligible pregnant women with GDM were randomized into two groups to receive a daily synbiotic capsule [500 mg of *L.acidophilus*(5 × 10^10^ CFU/g), *L.plantarum*(1.5 × 10^10^ CFU/g), *L.fermentum*(7 × 10^9^ CFU/g), *L.Gasseri*(2 × 10^10^ CFU/g) and 38.5 mg of fructo-oligo-saccharides], or placebo, for 6 weeks. The ratios of TC/HDL-C, LDL/HDL-C, and logTG/HDL-C were calculated as the atherogenic indices. Serum hs-CRP and MDA concentrations were quantified before and after the intervention. *Cohen’s d(d)* was used to calculate the magnitude of the effect.

**Results:**

Ninety participants completed the study. There was no significant difference in dietary antioxidant and mineral intakes between the two groups. Compared with placebo, synbiotic supplementation resulted in a significant decrease in logTG/HDL-C ratio with a medium–low effect size (mean difference = −0.11; 95% CI −0.21, 0; *P* values for the placebo and the intervention groups were 0.02, and 0.042, respectively; *P *between groups = 0.003; *d* = 0.25). No significant changes were observed in other parameters.

**Conclusions:**

Overall, 6 weeks of synbiotic supplementation in women with GDM resulted in a significant improvement in logTG/HDL-C, suggesting that synbiotics may have a beneficial role in reducing the risk of future CVDs associated with GDM. Nevertheless, more studies are needed to confirm the veracity of these results.

*Trial Registration* IRCT201511183140N16 (December 29th, 2015).

## Introduction

Gestational diabetes mellitus (GDM) is defined as any degree of glucose intolerance with the onset or first recognition during pregnancy [1]. According to the most recent (2017) International Diabetes Federation (IDF) estimates, GDM affects approximately 14% of pregnancies worldwide, but the figures vary depending on the demographic characteristics of the population [2]. It is well-known that GDM have negative consequences for both the mother and the offspring [3]. Insulin resistance may develop as the pregnancy advances into the third trimester due to additional hormones released during the pregnancy that might impair the efficacy of insulin and induce hyperglycemia [4]. This could increase the risks of gestational hypertension and preeclampsia, as well as the risks of type-2 diabetes (T2DM) and cardiovascular diseases (CVD) later in life [4]. According to a recent systematic review and meta-analysis, women with GDM had a twofold higher risk of future CVD compared to those who did not have GDM, which remained associated with a 56% higher risk of future cardiovascular events, even when restricted to women who did not develop T2DM [5]. Atherogenic indices, which generally include the ratios of total cholesterol (TC)/high-density lipoprotein cholesterol (HDL-C), low-density lipoprotein cholesterol (LDL-C)/HDL-C, and logarithm of triglycerides (TG)/HDL-C, are strong predictors of the risks of atherosclerosis and CVDs [6]. On the other hand, the role of inflammation and increased oxidative stress in the initiation and development of atherosclerosis and susceptibility to CVD is well established [7]. Gestational diabetes mellitus is demonstrably associated with increased levels of both inflammation and oxidative stress [8]. Insulin resistance causes an increase in blood high-sensitive C-reactive protein (hs-CRP) and malondialdehyde (MDA), which are important inflammatory and oxidative stress markers in women with GDM [9, 10]. Empirical evidence has demonstrated that elevated levels of hs-CRP and MDA are not only associated with increased blood glucose concentrations and adverse events during pregnancy [11, 12], but also are strong predictors of future cardiovascular events [13]. In fact, increased hs-CRP levels and oxidative stress markers are linked to insulin resistance and carotid intima-media thickness in patients with diabetes, all of which contribute to an increased cardiovascular risk in this population [14].

In recent decades, synbiotics have gained popularity due to their favorable effects on the gut microbiota. [15, 16]. A synbiotic is a combination of probiotics and prebiotics, most commonly oligosaccharides or inulin, which demonstrate an additive action to restore normal bacterial flora [17]. Evidence suggests that synbiotics may exert positive effects on alleviating inflammation and insulin resistance in patients with T2DM [18] and women with GDM [19], although the results are still controversial. Synbiotics may promote human health through lowering serum cholesterol, producing short chain fatty acids (SCFA), and increasing bile salt deconjugation [20]. However, randomized controlled trial (RCT) studies examining the benefits of synbiotics or probiotics on inflammatory and oxidative stress markers in pregnant women with GDM are rare [21, 22]. According to a recent systematic review, only three previous human investigations assessed the effects of synbiotics on hs-CRP and MDA levels in women with GDM with both significant and insignificant findings [19], highlighting the necessity of conducting additional research in this population. Furthermore, no previous clinical trial studies have evaluated the effects of synbiotics or probiotics supplementation on atherogenic indices in women with GDM, who are at a high risk of developing CVD. As a result, the current research examined the effect of synbiotic supplementation on atherogenic indices, hs-CRP, and MDA levels in pregnant women with GDM, all of which are major predictors of future CVD risk.

## Materials and methods

### Compliance with Ethical Standards

This is a secondary data-analysis of a previous study [23] that was conducted in accordance with the Ethics Committee of Tabriz University of Medical Sciences, Tabriz, Iran (No. TBZMED.REC.1394.688). The recruitment of participants was initiated in January, 2016. The details of the study were described to every participant by the main researcher. Every volunteer signed an informed consent form prior to participating. The present investigation was registered at the Iranian Registry of Clinical Trials with the code, IRCT201511183140N16, registered on December 29th, 2015 [24].

### Sample size and randomization

According to a previous study [23], sample size was computed using a 95% CI, a power of 80%, and anticipating a 15% dropout rate. The final sample size was estimated to be 45 participants in each intervention group. The homeostasis model assessment-insulin resistance (HOMA-IR) was used the key variable. Randomization was performed using random allocation software, and sealed envelopes were used for concealment of randomization. All of the participants and researchers were blinded throughout the study to the final analysis. After the statistical analysis was completed, code breaking was done by someone who was not aware of the study.

### Study design and participants

The present double-blind, placebo-controlled, RCT study was conducted at the Diabetes East Health Center in Ahwaz, Iran. Eligible participants were pregnant women between the ages of 18 and 40 (y) who were in weeks 24–28 of pregnancy and had GDM, according to the American Diabetes Association's criteria [25]. A 75 g oral glucose tolerance test (OGTT) was performed in a fasted condition and at 24–28 weeks of pregnancy. The diagnosis of GDM was then made when any of the following criteria was met: fasting plasma glucose ≥ 92 mg/dL, 1-h plasma glucose ≥ 180 mg/dL, and 2-h plasma glucose ≥ 153 mg/dL [26].

Participants were not included if they had lactose intolerance, pre-eclampsia or eclampsia, had placental abruption, any of the liver, kidney, inflammatory or immune deficiency diseases, as well as thyroid disorders, or used any kind of hormone replacement therapies, anti-diabetic medications, cholesterol-lowering drugs, antibiotics, or consumed any kind of synbiotics/probiotics products in the month before the diagnosis of GDM. If participants reported any evidence of gastro-intestinal side effects after taking the synbiotic tablets, they were excluded from the study.

Ninety-five pregnant women with GDM who met the inclusion criteria were randomly allocated into two groups to receive either synbiotic capsules (n = 48) or placebo capsules (n = 47). Finally, 90 women completed the study. Figure 1 shows the complete flow of the study based on the Consolidated Standards of Reporting Trials (CONSORT) flow diagram. Every participant was asked to take one capsule after lunch every day for six weeks, and they were not allowed to change their normal dietary intake or physical activity during the study.

**Fig. 1:** Flow of study

Both the synbiotic and placebo capsules (LactoFem) were provided by ZistTakhmir Pharmaceutical Company in Tehran, Iran. The contents in each synbiotic capsule were 500 mg of *Lactobacillus* probiotic strains [*L.acidophilus* (5 × 10^10^ CFU/g), *L.plantarum* (1.5 × 10^10^ CFU/g), *L.fermentum* (7 × 10^9^ CFU/g) and *L.Gasseri* (2 × 10^10^ CFU/g)]. The synbiotic supplements also contained 38.5 mg of fructo-oligo saccharides (FOS) and 300 mg of lactose as prebiotics, which help these bacteria grow. Other ingredients were colloidal silicon dioxide, magnesium stearate, and talc (each weighing 5.5 mg), as well as neutral flavorings and sweeteners. The placebo capsules had all the contents except for the probiotic strains, FOS and lactose. Consumption of magnesium stearate is generally considered safe at levels below 2500 mg/kg/day [27]. The probiotic and placebo capsules were similar in shape, taste, smell, and texture, and were labeled with specific codes (“A” or “B”). Sufficient allocated capsules were given to participants every 2 weeks. They were also asked to bring the remaining capsules with them to each visit. Compliance with consumption was monitored via phone calls and face-to-face interviews.

### Anthropometric and dietary intake measurements

Trained personnel performed anthropometric measurements. A portable stadiometer was used for the measurement of height nearest to 0.1 cm, and weight was measured with light clothing using a digital scale (Seca, Germany) nearest to 0.1 kg. Body mass index (BMI) was estimated by dividing weight (kg) by height (m^2^) based on participants’ pre-pregnancy weights. The pre-pregnancy weight was recorded based on the maternal report at the time of recruitment. If pre-pregnancy weight data was not available, the pre-pregnancy weight was estimated using Institute of Medicine (IOM) weight gain recommendations based on the pregnancy trimester (0.15 kg/week in trimester 1, and 0.42 kg/week in trimesters 2–3 for women with normal body weight, and 0.2–0.3 kg for women with overweight and obesity in trimesters 2–3) and subtracted from the participants’ measured weight on the interview day [28]. Dietary intake was measured using a 24-h food recall and the 3-day food record. Using household measures, the average intakes were converted to grams per day [29]. We used the Nutritionist-4 software program (First Databank, Hearst Corp, San Bruno, CA, USA), which was adapted for Iranian foods, to assess participants' dietary macro- and micronutrient intakes.

### Measurements of atherogenic Indices, serum hs-CRP and MDA concentration

Six ml of 10–12 h overnight fasting blood samples was drawn at the baseline and at the end of the intervention, which were centrifuged for 10 min at 2500 rpm (Beckman Avanti J-25; Beckman Coulter, Brea, CA, USA). Serums were immediately kept at 80 °C until analysis. The conventional enzymatic approach was used to determine serum TC, TG, HDL-C, and LDL-C. (Pars Azmun kit, Karaj, Iran). The values of atherogenic parameters, including the ratios of TC/ HDL-C, LDL-C/HDL-C, and log TG/HDL-C, were calculated based on previously published data [23]. Serum hs-CRP was assessed using the immunoturbidometry method. The thiobarbituric acid reactive substance spectrophotometric test was used to evaluate the plasma levels of MDA [30].

### Statistical methods

We used the statistical software package SPSS (version 22) for conducting all the statistical analyses. The quantitative variables were reported as mean ± standard deviation (SD). The Kolmogorov–Smirnov test was used to assess the normality of the distribution of the quantitative variables. At the beginning of the study, between-group comparisons of normal and non-normal quantitative variables were conducted using independent sample t-tests and Mann–Whitney U tests, respectively. For comparing data before and after the intervention within each group, paired student’s *t*-tests and Wilcoxon Signed Ranks Tests were used. Finally, analysis of covariance (ANCOVA) was used at the end of the study to compare between-group differences. The mean difference (MD) and confidence interval (CI) were finally reported. Covariates were considered to be age, BMI, energy intake and baseline measurements. Additionally, *Cohen’s d* effect size was estimated at the end of the study for all of the outcomes to measure the magnitude of the effect between groups, via estimating the difference between the means at post-intervention, divided by the pooled SD. Accordingly, effect sizes were defined as small (*Cohen’s d* = 0.2), medium (*Cohen’s d* = 0.5), and large (*Cohen’s d* = 0.8), which corresponded with the 58^th^, 69^th^, and 79^th^ percentiles of the distribution of the control group, respectively [31]. *P* < 0.05 was set as the statistical significance threshold.

## Results

As shown in the study flow diagram (Fig. 1), of the 95 eligible participants, 90 women completed the study to the final analyses [45 women in each group]. Five of the participants were withdrawn during the study (2 and 3 individuals in each placebo and synbiotic groups, respectively) due to miscarriage (n = 2), incomplete supplement consumption at the expected time (n = 1), and personal reasons (n = 2). There were no major side effects recorded after taking the synbiotic supplements.

Table 1 shows the baseline data of participants. Accordingly, we found no significant differences in the mean values of age, height, gestational week, pre-gestational weight, and gestational weight, at the initiation of the study between the two groups. Similarly, there were no significant differences between the groups at the baseline of the study in terms of macro- and micro-nutrient intakes, except for the energy intake [1880 (922, 2871) kcal in the synbiotic group *vs.* 1663.3 (821.9, 2550.1) kcal in the placebo group; *P* < 0.05].

**Table 1:** Participants’ baseline characteristics

Variables	Placebo group (n = 45)	Synbiotic group (n = 45)	P values
Demographic data^a^			
Age (years)	30.3 (5.6)	29.4 (5.8)	0.44
Height (cm)	160.2 (5.9)	161.3 (5.6)	0.38
Gestational age (weeks)	26.2 (2.3)	25.8 (1.8)	0.68
Anthropometric characteristics^a^			
Pre-gestational weight (kg)	68 (10.4)	63.9 (11.1)	0.09
Gestational weight at study baseline (kg)	72.1 (10.7)	69 (12.8)	0.14
Gestational BMI at study baseline (kg/m^2^)	28.2 (4.7)	26.4 (4.1)	0.06
Glycemic profile indices			
FPG at study baseline (mg/dl)^a^	85.8 (10.4)	90.5 (11.8)	0.06
Insulin at study baseline (µIU/ml)^b^	12.6 (8.1, 19.7)	11.7 (8.4, 21.7)	0.81
Dietary intakes^b^			
Energy (kcal/day)	1663.3 (821.9, 2550.1)	1880 (922, 2871)	0.02^a^
Calcium (mg/day)	543.6 (83.9, 1915.1)	778.1 (141.2, 1916.2)	0.32
Iron (mg/day)	15.6 (7.05, 35.1)	18.9 (9.25, 38.3)	0.31
Zinc (mg/day)	6.5 (2.2, 13.5)	7.1 (2.3, 16.1)	0.21
Vitamin A (mg/day)	304.4 (87.1, 2651.1)	301 (40.6, 2457.1)	0.51
Vitamin C (mg/day)	90.6 (1.2, 301.6)	99.5 (8.2, 300.4)	0.74

*BMI* body mass index; *FPG* fasting plasma glucose

^a^Data are presented as Mean (SD)

^b^Data are presented as median (25, 75 percentiles)

^c^Statistically significant (*P* < 0.05)

Based on the analyses, no significant changes were seen in the measures of TC [MD(CI) = 2.1 (− 10.4 to 14.6) mg/dL), LDL-C [MD(CI) = 0.06 (− 9.8 to 9.9) mg/dL] and TG [MD(CI) = 4.0 (− 13 to 21.2) mg/dL] at the end of the investigation, while within-group comparisons revealed a significant increase in HDL-C in the intervention group [MD(CI) = 5.1 (1.7–8.5) mg/dL], following the synbiotic supplementation [details of data are reported previously [23]]. Our findings also showed a significant decrease in logTG/HDL-C in the intervention group compared to the placebo group at the end of the study. However, a low-medium effect size was detected, which signified that almost 60% of the mean changes in logTG/HDL-C in the control group were below the mean measures in the intervention group [MD(CI) = −0.11 (−0.21, 0); *P* = 0.003; *Cohen’s d* = 0.25]. Within-group analysis also showed a significant decrease in logTG/HDL-C in the intervention group [MD(CI) = −0.05 (−0.09, 0.01)]. No significant differences were observed in other atherogenic indices, including the ratios of TC/HDL-C and LDL-C/HDL-C, at the end of the study (Table 2).

**Table 2:** Changes in atherogenic indices, hs-CRP and MDA levels at the baseline and at after the 6 weeks of synbiotic supplementation

Variable	Period	Placebo group (n = 45)	Synbiotic group (n = 45)	MD (95% CI)^a^ between groups	*P* value	Effect Size *(Cohen’s d)*^b^
MDA (μmol/L)	Initial	1.78 (0.45)	1.82 (0.82)	0.04 (−0.24, 0.32)	0.78	
	End	1.77 (0.46)	1.89 (0.42)	0.12 (−0.05, 0.29)	0.28	0.16
	MD (95% CI) within groups^c^	0.01 (−0.16 to 0.15)	0.07 (−0.15 to 0.29)			
	*P* value	0.9	0.49			
hs-CRP (μg/mL)	Initial	5.17 (2.47, 7.46)	4.52 (2.9, 11.4)	−0.92	0.57	
	End	5.9 (3.1, 8.3)	4.4 (2.68, 11.35)	−1.5	0.66	0.11
	Median difference	0.73	−0.12			
	*P* value	–	–			
TC/HDL-C	Initial	4.26 (1.25)	4.46 (1.95)	0.2 (−0.49, 0.88)	0.58	
	End	4.45 (1.19)	4.18 (1.25)	−0.27, −0.78, 0.24)	0.06	0.12
	MD(95% CI) within groups^c^	0.19 (−0.18, 0.54)	−0.28 (−0.75, 0.2)			
	*P* value	0.31	0.25			
LDL-C/HDL-C	Initial	2.54 (0.87)	2.73 (1.6)	0.19 (−0.36, 0.73)	0.73	
	End	2.62 (0.88)	2.45 (0.96)	−0.17 (−0.56, 0.22)	0.06	0.1
	MD(95% CI) within groups^c^	0.08 (−0.22, 0.36)	−0.28 (−0.76, 0.2)			
	*P* value	0.59	0.19			
logTG/HDL-C	Initial	0.48 (0.25)	0.48 (0.28)	0.001 (−0.11, −0.15)	0.97	
	End	0.55 (0.26)	0.43 (0.25)	−0.11 (−0.21, 0)	**0.003**	0.25
	MD(95% CI) within groups^c^	0.07 (0.02, 0.12)	−0.05 (−0.09, 0.01)			
	*P* value	**0.02**	**0.042**			

*MD* mean differences, *MDA* malondialdehyde, *hs-CRP* high-sensitivity C-reactive protein, *TC* total cholesterol, *HDL-C* high density of lipoprotein cholesterol, *LDL-C* low-density of lipoprotein cholesterol, *TG* triglycerides

Bold values indicate statistically significance (*P* < 0.05)

Data are shown as mean (SD); data for hs-CRP are presented as median (25, 75 percentiles)

^**a**^Independent student t-tests were used at beginning of the study for between-group comparison, except for hs-CRP measures which was estimated by Mann–Whitney U-tests. At the end of the study, differences between groups were assessed using analysis of covariance (ANCOVA) adjusted for baseline values, age, BMI and energy intake

^**b**^*Cohen’s d* values, were defined as the difference between the means after the intervention, divided by the pooled SD. *Cohen’s d* of 0.2, 0.5 and 0.8 locate at 58th, 69th and 79th percentile of the distribution of the control group, respectively

^**c**^Paired student t-tests were used for within-group comparisons, except for hs-CRP measures which was estimated by non-parametric Wilcoxon signed ranks tests

Concerning hs-CRP and MDA levels, between-group analyses reported no significant alterations in the mentioned parameters after the synbiotic supplementation (*P* > 0.05) (Table 2).

## Discussion

The key findings of the present study indicated that pregnant women diagnosed with GDM who consumed synbiotics for 6 weeks had a lower ratio of logTG-HDL-C, as the main atherogenic index, compared to the placebo group. However, there were no substantial differences in hs-CRP and MDA levels in the intervention group compared to the control group after the synbiotic supplementation.

To our knowledge, no previous clinical trial study has assessed the effect of synbiotic or probiotic supplementation on atherogenic indices in women with GDM. Only one study by Ejtahed, et al. evaluated the effect of yogurt enriched with probiotics in patients with T2DM, and, consistent with our findings, the authors reported a significant decrease in logTG/HDL-C ratio [32]. Although Ejtahed et al., showed promising effects of probiotics on the atherogenic index, they used yogurt as the probiotic carrier instead of probiotic supplements [32]. Previous evidence suggests that the presence of other nutrients such as calcium, sphingolipids, and protein in dairy products enriched with probiotics can have positive effects on CVD [33], suggesting that the efficacy of dairy products enriched with probiotics on atherogenic indices may not be significant enough to introduce synbiotics or probiotics as CVD-preventive agents, the findings of our study on synbiotic supplements’ single favorable effect on the atherogenic index would be more noteworthy.

The precise mechanisms by which synbiotics benefit atherogenic indices are unknown, but can be attributed to the positive correlation between probiotics and serum HDL-C concentrations [34]. In fact, HDL-C transports cholesterol in the form of cholesteryl esters to the liver for further hydrolysis [35]. It has been proposed that probiotics or synbiotics lower cholesterol levels by changing cholesteryl esters and lipoprotein transporter pathways [36]. We previously reported a considerable increase in serum HDL-C concentrations after synbiotic supplementation in women with GDM [23], which could be the major rationale for the current significant improvement in logTG/HDL-C as the main atherogenic measure. Similarly, a meta-analysis also highlighted that an increase in HDL-C concentrations is strongly associated with a reduced risk of CVD compared with changes in blood TG levels [37].

Despite several human studies evaluating the effects of probiotics or synbiotics on inflammatory or oxidative stress markers in different populations, including patients with T2DM [38, 39], only a few clinical trial studies with inconsistent findings have evaluated this association in pregnant women with GDM [40, 41]. Concordant with our results, Taghizadeh et al. [41] showed that synbiotic food enriched with *Lactobacillus sporogenes* (1 × 10^7^ CFU) in 52 pregnant women with GDM, during their third trimester, had no significant impact on hs-CRP levels after 9 weeks. Other studies also found that giving probiotic supplements to T2DM patients for 6 weeks [38] or 12 weeks [42], did not change serum levels of hs-CRP or MDA. Due to the low number of RCTs studying the relationship between probiotics and diabetes mellitus, only a few meta-analyses have been published in this topic [43–45]. A recent meta-analysis of RCTs that assessed the effects of probiotic and synbiotic supplementation on inflammatory markers, revealed that the levels of hs-CRP decreased significantly following synbiotic supplementation in patients with metabolic disorders, and arthritis, while no meaningful changes were reported in patients with other health conditions including GDM. Another meta-analysis of four studies found that probiotic supplementation reduced MDA levels in patients with GDM, though the authors claimed that the data was insufficient to determine the final magnitude of the effects [19]. Above all, there is insufficient information on the anti-inflammatory and antioxidant effects of probiotics in women with GDM, and the results are inconsistent, which could be related to differences in study designs, strain-specificities of these microorganisms, and probiotic doses and durations. Furthermore, the current non-significant changes in hs-CRP and MDA levels in women with GDM could be explained by the normal range of these parameters among participants at the start of the study, preventing probiotic supplementation from having a major impact on these markers.

Although the exact mechanisms by which synbiotics and probiotics supplementation have possible beneficial effects on hs-CRP and MDA levels [21, 46] are unknown, evidence has demonstrated several putative mechanisms, including decreasing gut dysbiosis and intestinal leakage, which reduces the development of inflammatory biomarkers [47], as well as the production of SCFAs, which blocks the enzymatic synthesis of hepatic CRP [48]. Meanwhile, as previously indicated, research into the effects of dairy products containing probiotic bacteria has yielded additional promising results. This could be due to the high calcium and natural bioactive content of probiotic dairy products [49], highlighting the need for more research into the anti-inflammatory, anti-oxidant, and CVD-protective effects of synbiotic or probiotic supplements alone, particularly in GDM patients.

The present investigation has many strengths. This study reported the effects of synbiotics on atherogenic indices, hs-CRP and MDA, as the most important predictors of future CVD risk in women with GDM, who are at a higher risk of future CVD. We used a statistically justified sample size, compared with previous similar studies that did not provide such justification [21, 41]. In addition, the *Cohens' d* effect sizes were estimated to evaluate the magnitude of the effects, in addition to performing basic analyses and determining the significance of final conclusions based on *P* values. Moreover, in our study, we restrained all the participants from taking foods or supplements that contained either probiotics or synbiotics, allowing us to assess the sole administration of synbiotic supplementation. Furthermore, we used almost all of the available probiotic bacteria and administered active probiotic capsule supplements, which are reported to have better functions in the host body [50]. We also included pregnant women with GDM who were not on insulin therapy, as any existing treatment for gestational diabetes could interfere with synbiotic efficacy or affect the composition of gut microbiota [51]. Despite the strengths of the present study, some limitations should also be mentioned. We were unable to conduct a longer intervention period, mostly due to the pregnancy status of participants. Stool samples were not also assessed to evaluate the microbial composition of the gut and feces. Moreover, due to budget limitations, we did not investigate other critical biochemical indicators predicting future CVD risks in this population.

## Conclusions

This RCT investigated the effectiveness of synbiotic supplementation on atherogenic indices, along with hs-CRP and MDA levels, as potential predictors of future CVD risk, among women with GDM. The principal findings from this study suggested that the pregnant women who consumed synbiotic supplements for 6 weeks had a lower ratio of logTG/HDL-C, than those who took placebo. Following synbiotic treatment, no significant changes in hs-CRP and MDA levels were found. The significant reduction in logTG/HDL-C, an important atherogenic measure, implies that synbiotics may have a CVD-preventive effect in pregnant women with GDM who are at a higher risk of future CVD. However, since the changes in logTG/HDL-C were so minor and because there is a lack of potential previous findings pertaining to the exact CVD-preventive role of synbiotic supplementation among women with GDM, more studies, with longer duration and various supplement dosages, are still needed to confirm the veracity of these results.

## Data Availability

Not applicable.

## Abbreviations

GDM: Gestational diabetes mellitus
T2DM: Type-2 diabetes mellitus
CVD: Cardiovascular disease
hs-CRP: High-sensitivity C-reactive protein
MDA: Malondialdehyde
CFU: Colony forming unit
TG: Triglycerides
TC: Total cholesterol
HDL-C: High density lipoprotein cholesterol
LDL-C: Low-density of lipoprotein cholesterol
BMI: Body mass index
SCFA: Short-chain fatty acids
FPG: Fasting plasma sugar
OGTT: Oral glucose tolerance test
FOS: Fructo-oligo saccharides
MD: Mean difference
CONSORT: Consolidated standards of reporting trials
